The article "Semi-Supervised Multi-View Clustering with Weighted Anchor Graph Embedding" was published in 2021. Journal: Comput Intell Neurosci.

# Semi-Supervised Multi-View Clustering with Weighted Anchor Graph Embedding

**DOI:** 10.1155/2021/4296247

**Published:** 2021-07-26

**Authors:** Senhong Wang, Jiangzhong Cao, Fangyuan Lei, Qingyun Dai, Shangsong Liang, Bingo Wing-Kuen Ling

**Affiliations:** ^1^School of Information Engineering, Guangdong University of Technology, Guangzhou 510006, China; ^2^Guangdong Provincial Key Laboratory of Intellectual Property and Big Data, Guangdong Polytechnic Normal University, Guangzhou 510006, China; ^3^School of Computer Science and Engineering, Sun Yat-sen University, Guangzhou 510006, China

## Abstract

A number of literature reports have shown that multi-view clustering can acquire a better performance on complete multi-view data. However, real-world data usually suffers from missing some samples in each view and has a small number of labeled samples. Additionally, almost all existing multi-view clustering models do not execute incomplete multi-view data well and fail to fully utilize the labeled samples to reduce computational complexity, which precludes them from practical application. In view of these problems, this paper proposes a novel framework called Semi-supervised Multi-View Clustering with Weighted Anchor Graph Embedding (SMVC_WAGE), which is conceptually simple and efficiently generates high-quality clustering results in practice. Specifically, we introduce a simple and effective anchor strategy. Based on selected anchor points, we can exploit the intrinsic and extrinsic view information to bridge all samples and capture more reliable nonlinear relations, which greatly enhances efficiency and improves stableness. Meanwhile, we construct the global fused graph compatibly across multiple views via a parameter-free graph fusion mechanism which directly coalesces the view-wise graphs. To this end, the proposed method can not only deal with complete multi-view clustering well but also be easily extended to incomplete multi-view cases. Experimental results clearly show that our algorithm surpasses some state-of-the-art competitors in clustering ability and time cost.

## 1. Introduction

In many practical applications, a growing amount of real-world data naturally appears in multiple views, which are called multi-view data, where the data may be characterized by different attributes or be collected from diverse sources. For example, an image can be described with different features, such as SIFT (Scale-Invariant Feature Transform), HOG (Histogram of Oriented Gradient), LBP (Local Binary Pattern), etc. [1]; a piece of specific news can be reported to multiple news organizations [2]; and a web page can be represented as a web page with links, texts, and images, respectively [3]. In other words, all of these objects are characterized by different characteristics, and each characteristic is referred to as one view describing the object. Generally, an individual view has a wealth of information to execute machine learning tasks, but it ignores leveraging the consistent and complementary information from multiple views [4]. Proper use of such information has the possibility of elevating various machine learning performances. Therefore, it is critical to consider how to effectively leverage such information.

Multi-view clustering, which adaptively separates data into corresponding groups by utilizing the consistency or complementarity principle among multiple views, is a very popular research direction. From the perspective of involved technologies, most of the existing literature reports are roughly classified into three types: matrix factorization-based, graph-based, and subspace-based approaches. As Kang et al. [5] pointed out, matrix factorization-based approaches seek a common matrix among different views, and graph-based approaches explore a common affinity graph, while subspace-based approaches learn the consensus subspace with low dimension. Therefore, as multi-view clustering, the key to obtaining high performance is to confirm that the optimal consistent representation is generated. To this end, multiple multi-view clustering models have been presented [6–17] and widely used in various real-world scenarios, for instance, object recognition [18], feature selection [19], information retrieval [20], etc.

One of the basic assumptions is that all views are complete, which is adopted by the aforementioned multi-view clustering approaches. However, in real-world applications, it is very common that samples are missing in some views for a lot of reasons, such as man-made faults or temporary failure of the sensor. Thus, previous complete multi-view methods cannot work well in this scenario since the pairwise information of samples missing some views cannot be directly used. If we want to apply conventional multi-view clustering algorithms to deal with the incomplete dataset, we can either remove the samples with incompleteness or fill incomplete samples with information during pre-processing. Nevertheless, these pre-processing methods will cause the original data to lose information or introduce noise, which makes conventional multi-view clustering methods unavoidably degrade or even fail. Therefore, incomplete multi-view clustering cases have drawn increasing interest recently, and many attempts have been made to tackle this problem [2, 21–26].

Moreover, real-world data usually contains a small number of labeled samples in some practical applications. The aforementioned methods are unsupervised and cannot leverage prior information to improve the performance, which limits their application. In practice, labeled samples are available, and efficiently exploiting these data can significantly improve clustering performance and reduce clustering time consumption. Inspired by this framework, some advanced semi-supervised multi-view clustering frameworks have recently been created to perform various clustering tasks [27–33]. However, most of these methods learn the optimal common indicator matrix from multiple views by performing alternative optimization algorithms, which leads to high computational complexity and cannot be widely used.

In view of the above issues, we present a new framework called Semi-supervised Multi-View Clustering with Weighted Anchor Graph Embedding (SMVC_WAGE), which is conceptually simple and efficiently generates high-quality clustering results in practice. SMVC_WAGE employs inherent consistency and external complementary information to seek the optimal fusion graph that spans multiple views compatibly in structure. Specifically, we apply the anchor graph learning to bridge all the intrinsic view samples, which can greatly enhance efficiency and improve stableness. Moreover, this can also solve the dilemma that samples sharing no common views cannot be directly used for computing cross-view similarities. Besides, instead of regularizing or weighting the loss of each view in a conventional way, the proposed method directly combines the graphs of different views to construct the global optimal fused graph, where the weights are learned in a nearly parameter-free manner. Therefore, through exploring anchor selection strategy from labeled samples and designing the weighted fusion mechanism for multiple views simultaneously, the proposed method can not only deal with complete multi-view clustering well, but also be easily extended to the incomplete multi-view instance. The main contributions of this paper are summarized as follows:

1. We provide a simple and effective anchor strategy. Based on these anchor points, the proposed method can exploit the intrinsic and extrinsic view information to bridge all samples and capture more reliable nonlinear relations, which can greatly enhance efficiency and improve stableness while partitioning multi-view data into different clusters.
2. We propose a novel graph fusion mechanism that constructs the global fused graph via directly coalescing the view-wise graphs, and the procedure is nearly free of parameters.
3. We present a more general semi-supervised clustering framework that can deal with complete multi-view clustering well and be easily extended to incomplete multi-view cases.
4. Experimental results on six widely used multi-view datasets clearly show that our algorithm surpasses some state-of-the-art competitors in clustering ability and time cost.

Other parts of the paper are organized as follows: Section 2 briefly reviews the related works. In Section 3, the proposed algorithm is described in detail. Afterwards, the experimental results and discussion are given in Section 4. Finally, Section 5 concludes the paper.

## 2. Related Work

In this section, we firstly make an introduction of recent progress of two specific multi-view clustering approaches. Then, we briefly describe the related work of semi-supervised multi-view clustering.

### 2.1. Complete Multi-View Clustering

Multi-view clustering exploits the consistent and complementary information from multi-view data to increase clustering performance and stability, which has attracted extensive attention recently. Numerous multi-view clustering models have been built. Usually, the multi-view clustering approaches assume that total samples have complete information in each view, where the samples are called complete multi-view data. Roughly speaking, in terms of related techniques, they can be mainly divided into two sections: graph-based and subspace-based methods.

Graph-based methods aim to construct the optimal fusion graph which is performed by graph-cut or other techniques to obtain the final result. Li et al. [6] developed a novel approach, named Multi-view Spectral Clustering (MVSC), which selects several uniform salient points to construct a bipartite graph that represents the manifold structures of multi-view data. Nie et al. [7] offered a new approach called Self-weighted Multi-view Clustering (SwMC), which is completely self-weighted and directly assigns the cluster label to the corresponding data point without any post-processing. Wang et al. [8] proposed a general Graph-based Multi-view Clustering (GMC), which jointly learns the graph of each view and the unified graph in a mutually enhanced manner and directly generates the final clustering result. Tang et al. [9] presented a robust model for Multi-view Subspace Clustering, which designs a diversity regularization term to enhance the diversity and reduce the redundancy among different feature views. Additionally, graph-based methods usually need to predefine graphs, and the quality of the graph largely determines the final clustering performance. The work in [10] introduced a novel model named Multi-view Clustering with Graph Learning (MVGL), which learns one global graph from different graphs constructed by all views to promote the quality of the final fusion graph. The work in [11] presented a novel method named Multi-view Consensus Graph Clustering (MCGC), which minimizes disagreement among all views and imposes a low-rank restraint on the Laplacian matrix to gain a unison graph. The study in[12] proposed a novel model called Graph Structure Fusion (GSF), which designs an objective function to adaptively tune the structure of the global graph. The work in [13] proposed a novel multi-view clustering method, which learns a unified graph via cross-view graph diffusion (CGD), where the initial value entered is each predefined view-wise graph matrix. To further learn a compact feature representation, the study in [14] proposed to capture both the shared information and distinguishing knowledge across different views via projecting each view into a common label space and preserve the local structure of samples by using the matrix-induced regularization.

Subspace-based methods are widely studied; they utilize various techniques to obtain low-dimensional embedding. In general, they can efficiently reduce the dimensionality of the raw data and be easy to explain. Because of this property, the study in [15] proposed to simulate different views as different relations in a knowledge graph, which learns a unified embedding and several view-specific embeddings from similarity triplets to perform multi-view clustering. The work in [16] proposed a novel model called Latent Multi-view Subspace Clustering (LMSC), which encodes complementary information between different views to automatically learn one latent consistent representation. To decrease the computational complexity and this memory requirement, the work in [17] introduced a novel framework entitled Binary Multi-View Clustering (BMVC), which jointly learns these collaborative binary codes and binary cluster structures to perform large-scale multi-view clustering.

### 2.2. Incomplete Multi-View Clustering

In practical applications, we are more likely to be provided with incomplete multi-view data. However, conventional multi-view clustering approaches unavoidably degrade or even fail while dealing with incomplete multi-view data. Recently, many works have been executed to solve this issue, which can be generally classified into matrix factorization-based and graph-based methods in terms of involved techniques.

Matrix factorization-based methods directly learn a latent consistent representation with low dimensionality from all views by utilizing the matrix factorization techniques. Li et al. [21] developed a pioneering approach called Partial multi-View Clustering (PVC), which learns a latent consistent subspace of complete samples and a private latent representation of incomplete samples by exploiting nonnegative matrix factorization (NMF) and sparsity norm regularization. Zhao et al. [22] presented a model that learns the compact global structure over the entire samples across all views by integrating Partial multi-View Clustering and graph Laplacian term. Shao et al. [23] presented the framework named Multi-Incomplete-view Clustering (MIC), which exploits weighted NMF and *L*_2,1_-norm regularization to learn the latent consistent feature matrix. Hu and Chen [24] proposed the approach called Doubly Aligned Incomplete Multi-view Clustering (DAIMC), which can handle negative entries through integrating weighted semi-NMF and *L*_2,1_-norm regularized regression. While the above approaches can deal with incomplete multi-view data, the comparatively large storage and computational complexities limit their real-world applications. Liu et al. [25] proposed a novel framework called Late Fusion Incomplete Multi-view Clustering (LF-IMVC), which simultaneously imputes each incomplete sample and learns a consistent indicator matrix.

Graph-based methods focus on learning the low-dimensional representation from each graph which is constructed by each view and uncover the relationships between all samples. Wen et al. [26] introduced a general framework, which learns the low-dimensional representations from all views via exploiting spectral constraint and coregularization term. Guo and Ye [2] proposed a new algorithm named Anchor-based Partial Multi-view Clustering (APMC), which integrates the intrinsic and extrinsic view information into the fused similarities via anchors; then, the unified clustering outcome can be achieved by performing spectral clustering on the fused similarities.

### 2.3. Semi-Supervised Multi-View Clustering

Semi-supervised multi-view clustering, which uses a small proportion of labeled samples as well as a great number of unlabeled samples to perform clustering, is one of the hottest research directions in machine learning. As the most popular technique in the area of semi-supervised multi-view clustering, graph-based methods construct a graph, where vertices contain unlabeled and labeled data and edges reflecting the similarity of vertices spread information from labeled to unlabeled vertices. Thinking of each kind of feature as a modality, Cai et al. [27] proposed an algorithm named Adaptive Multi-Modal Semi-Supervised classification (AMMSS), which jointly learns the weight and the commonly shared class indicator matrix. Karasuyama and Mamitsuka [28] proposed a new method called Sparse Multiple Graph Integration (SMGI), which linearly combines multiple graph Laplacian matrices with sparse weights for label propagation. Nie et al. [29] presented a new framework called Auto-weighted Multiple Graph Learning (AMGL), which automatically learns a set of optimal weights without any parameters. Nie et al. [30] presented a novel model named Multi-view Learning with Adaptive Neighbors (MLAN), which directly partitions the final optimal graph into corresponding groups and the process only has the parameter for the robustness. To take advantage of the information in multi-view data, Nie et al. [31] proposed a new model called Adaptive MUlti-view SEmi-supervised (AMUSE), which obtains a more suitable unified graph for semi-supervised learning via imposing a structural regularization term constraint. Aiming at the incomplete multi-view issue, Yang et al. [32] proposed a novel framework called Semi-supervised Learning with Incomplete Modalities (SLIM). It employs the inherent modal consistency to learn discriminative modal predictors and performs clustering via the external complementary information of unlabeled data. However, graph-based approaches do not always make sure whether the final representation has the same label as the raw data. Cai et al. [33] introduced a new semi-supervised Multi-View Clustering method based on Constrained Nonnegative Matrix Factorization (MVCNMF). It propagates the label information to a consistent representation via exploiting matrix factorization techniques.

## 3. Proposed Method

In this section, we elaborate our simple yet effective approach called Semi-supervised Multi-View Clustering with Weighted Anchor Graph Embedding (SMVC_WAGE), which provides a general framework for semi-supervised multi-view clustering. Specifically, SMVC_WAGE firstly provides a simple and effective anchor strategy that exploits the intrinsic and extrinsic view information to bridge all samples and capture more reliable nonlinear relations. Then, the proposed method learns the weight for each view via utilizing the seed-based semi-supervised *K*-Means and the designed mathematical techniques to seek the optimal fusion graph that spans multiple views compatibly in structure. Ultimately, spectral clustering is conducted on the global fused graph to obtain a unified clustering result. To this end, in the following, we describe the notation and problem definition firstly and then introduce the Semi-supervised *K*-Means based on Seed for single-view clustering. Thirdly, we propose SMVC_WAGE for solving both complete and incomplete multi-view clustering.

### 3.1. Notation and Problem Definition

1. *Notations*. Except in some specified cases, italic, not bold letters (*v*, *V*,…, ) represent scalars. Bold uppercase letters (**X**,…, ) denote matrices, while bold lowercase letters (**x**,…, ) are vectors. **I** is an identity matrix with an appropriate size, and **1** is an all-one vector with a compatible length.
2. *Definition*. As multi-view data, each sample is characterized by multiple views with one unified label. Assume that we are provided with a dataset *𝒳* = {**X**^(1)^, **X**^(2)^,…, **X**^(*V*)^} composed of *N* samples from the *V* views in *K* clusters, in which **X**^(*v*)^ = [**x**_1_^(*v*)^; **x**_2_^(*v*)^; …; **x**_*n*_^(*v*)^] ∈ ℝ^*n*×*d*_*v*_^ is the data matrix of the *v*-th view. Denote **x**_*i*_^(*v*)^ ∈ ℝ^*d*_*v*_^ as the *i*-th sample **x**_*i*_ in the *v*-th view, where *d*_*v*_ is the dimensionality of data features in the *v*-th view.

Multi-view clustering aims to classify all samples into *K* batches via utilizing the consistent and complementary information from multi-view data, where *K* is assumed to be predefined by users.

### 3.2. Semi-Supervised *K*-Means Based on Seed

The proposed method performs spectral clustering on the global fused graph to obtain a unified clustering result whereas *K*-Means clustering is the important component of spectral clustering. Additionally, for our method, the seed-based semi-supervised *K*-Means is the key step to learn the weights from multiple views. Therefore, it is necessary to review Semi-supervised *K*-Means based on Seed.

Without any loss of generalization, we assume a single-view data matrix **X** = [**x**_1_; **x**_2_; …; **x**_*n*_] ∈ ℝ^*n*×*d*^, where **X** can be acquired from the above-mentioned multi-view data. Suppose that the single-view data matrix **X** is categorized into *K* clusters {**C**_*l*_}_*l*=1_^*K*^. In a semi-supervised single-view clustering framework, we customarily collect a small amount of labeled data **X**_*S*_, termed the seed set **X**_*S*_⊆**X**, through prior knowledge, and we suppose that, for each cluster **C**_*l*_⊆**X**, there is typically at least one seed point **x**_*i*_ ∈ **X**_*S*_. Note that we take a disjoint *K* partitioning {**X**_*S*,*l*_}_*l*=1_^*K*^ of the seed set **X**_*S*_, so that **x**_*i*_ ∈ **X**_*S*,*l*_ belongs to **C**_*l*_. In semi-supervised *K*-Means, the seed set **X**_*S*_ is utilized to initialize the *K*-Means approach. Thus, the centroid of the *l*-th cluster **C**_*l*_ is initialized with the mean of the *l*-th partition **X**_*S*,*l*_; then, the semi-supervised *K*-Means objective function can be written as

(1) $$\begin{array}{c} J_{K-\text{ Means}}=\sum_{l=1}^{K}\sum_{i=1}^{N}{\left\|x_{i}-u_{l}\right\|}^{2}\delta \left(x_{i}-u_{l}\right), \end{array}$$

where **x**_*i*_ ∈ ℝ^*d*^ is the *i*-th sample **x**_*i*_ from the single-view data matrix **X**, **u**_*l*_ ∈ ℝ^*d*^ is the mean of the *l*-th partition **X**_*S*,*l*_, and *δ* is the Dirac delta function. Furthermore, **u**_*l*_ and *δ*(**x**_*i*_ − **u**_*l*_) can be defined as the following equations, respectively.

(2) $$\begin{array}{c} u_{l}=\frac{1}{\left|X_{S,l}\right|}\sum_{x\in X_{S,l}}x, \end{array}$$

(3) $$\begin{array}{c} \delta \left(x_{i}-u_{l}\right)=\left\{\begin{array}{cc} 1, & \text{if }l=\underset{h}{\arg\min}{\left\|x_{i}-u_{h}\right\|}^{2}\forall h\in \left[1,K\right],\\ 0, & \text{otherwise,} \end{array}\right. \end{array}$$

where |**X**_*S*,*l*_| is the number of samples in **X**_*S*,*l*_.

Through further analysis of *K*-Means objective function equation (1), its optimal solution is an NP-hard problem [34]. However, the objective function is quickly locally minimized and converges to a local optimum by using the efficient iterative relocation algorithms [35].

### 3.3. The Proposed Method for Complete Multi-View Data

#### 3.3.1. Anchor-Based Global Fused Similarity Matrix Construction in Multi-View Data

In recent years, some studies [2, 36, 37] apply an anchor-based scheme to form the similarity matrix **S**. Generally, the anchor-based scheme mainly consists of two steps. The first step is that *m* anchor points can be searched from the raw data, where *m* ≪ *n*. The second is that a matrix **Z** ∈ ℝ^*n*×*m*^ is designed to measure the similarity between anchor points and data points.

There are two common methods for anchor point generation: random selection and *K*-Means method. Random selection is to extract a portion of data as anchor points via adopting random sampling from original data. Although the random selection strategy saves time, it cannot ensure that the selected anchor points are always good, which makes the results neither ideal nor stable. *K*-Means approach utilizes the clustering centroids as anchor points, which makes the chosen anchors more representative in comparison with random selection. Nevertheless, an inevitable problem is that *K*-Means is sensible to its origin centroid. To eliminate this problem, the *K*-Means method requires numerous independent and repeated running. For this reason, exploiting the *K*-Means as a pre-processing or post-processing framework is also unpredictable and has computational complexity. Considering that several real samples may have the label in practice and real samples that belong to the same cluster have similar statistical characteristics, while samples belonging to different clusters have greater differences in statistical characteristics, we can obtain the seed set ${𝒳}_{𝒮}=\left\{X_{S}^{\left(1\right)},X_{S}^{\left(2\right)},\ldots ,X_{S}^{\left(V\right)},\hat{y}\right\}$ from the labeled samples in *V* views, where **X**_*S*_^(*v*)^ = [**X**_*S*,1_^(*v*)^; **X**_*S*,2_^(*v*)^; …; **X**_*S*,*K*_^(*v*)^] ∈ ℝ^*q*×*d*_*v*_^ denotes the seed set in the *v*-th view with *K* clusters, $\hat{y}=\left[{\hat{y}}_{1};{\hat{y}}_{2};\ldots ;{\hat{y}}_{q}\right]\in {\mathbb{R}}^{q}$ denotes the corresponding label vector, and *q* = |**X**_*S*_^(*v*)^| denotes the number of labeled samples. Then, the mean of each partitioning in the seed set *𝒳*_*𝒮*_ can be chosen as anchor points.

Specifically, the generated anchor points set in the *v*-th view can be represented as **U**^(*v*)^ = [**u**_1_^(*v*)^; **u**_2_^(*v*)^; …; **u**_*K*_^(*v*)^] ∈ ℝ^*K*×*d*_*v*_^, where **u**_*l*_^(*v*)^ can be obtained according to (2). Then, the similarity between data point **x**_*i*_^(*v*)^ and anchor point **u**_*l*_^(*v*)^ is defined as

(4) $$\begin{array}{c} Z^{\left(v\right)}=\frac{\exp\left(-D^{2}\left(x_{i}^{\left(v\right)},u_{l}^{\left(v\right)}\right)/\sigma^{2}\right)}{\sum_{l=1}^{K}\exp\left(-D^{2}\left(x_{i}^{\left(v\right)},u_{l}^{\left(v\right)}\right)/\sigma^{2}\right)}, \end{array}$$

where *𝒟*(**x**_*i*_^(*v*)^, **u**_*l*_^(*v*)^) is a distance function, such as *l*_2_ distance. The truncated similarity matrix **Z**^(*v*)^ ∈ ℝ^*N*×*K*^ is defined in *v*-th view based on a kernel function *𝒦*_*σ*_(·), and Gaussian kernel *𝒦*_*σ*_(**x**_*i*_^(*v*)^, **u**_*l*_^(*v*)^) = exp(−*𝒟*^2^(**x**_*i*_^(*v*)^, **u**_*l*_^(*v*)^)/*σ*^2^) is usually adopted. The parameter *σ* can be set to 1 without loss of generality.

For multi-view clustering, there is a common assumption that it can increase clustering performance and stability via appropriately exploiting the consistent and complementary information between different views. Based on this assumption, how to seamlessly combine multiple views is crucial to the final clustering result. Considering the differences in the clustering quality of each view, we first calculate the clustering accuracy of each view through the prior information and then obtain the weights for different views, where the view with greater clustering accuracy has larger weight during information fusion, and similarly the view with less clustering accuracy has a smaller weight. More specifically, we utilize the semi-supervised *K*-Means to acquire clustering result ${\hat{c}}^{\left(v\right)}=\left[{\hat{c}}_{1}^{\left(v\right)};{\hat{c}}_{2}^{\left(v\right)};\ldots ;{\hat{c}}_{q}^{\left(v\right)}\right]\in {\mathbb{R}}^{q}$ in the *v*-th seed set **X**_*S*_^(*v*)^, where anchor points set **U**^(*v*)^ of the *v*-th view is used to initialize semi-supervised *K*-Means. Note that ${\hat{c}}^{\left(v\right)}$ and $\hat{y}$ are the cluster labels and the ground-truth labels of the seed set **X**_*S*_^(*v*)^, respectively, and then we calculate the clustering accuracy of each view by (17) in the seed set *𝒳*_*𝒮*_. Furthermore, to ensure that the view with greater clustering accuracy has a larger weight, we apply the softmax function to acquire the weights for different views. The weights of the views can be represented by

(5) $$\begin{array}{c} w_{v}=\frac{e^{\lambda a_{v}}}{\sum_{j=1}^{V}e^{\lambda a_{j}}},\;\forall v\in \left[1,V\right], \end{array}$$

where **w**_*v*_ is the non-negative normalized weight for the *v*-th view and the sum of all elements of **w** is 1, **a**_*v*_ is the clustering accuracy for the *v*-th view in the seed set **X**_*S*_^(*v*)^, and *λ* is a scalar used to control the distribution of weights between different views.

The truncated similarity matrix **Z**^(*v*)^ can be obtained by (4), and then all truncated similarity matrices are integrated into a global truncated similarity matrix **Z** ∈ ℝ^*N*×*K*^ between all samples and anchors.

(6) $$\begin{array}{c} Z=\sum_{v=1}^{V}w_{v}Z^{\left(v\right)}. \end{array}$$

Once we obtain the matrix **Z**, the global fused similarity matrix **S** ∈ ℝ^*N*×*N*^ between all samples can be approximated by an anchor graph [36].

(7) $$\begin{array}{c} S=Z\Lambda^{-1}Z^{T}, \end{array}$$

where **Λ** = diag(**Z**^**T**^**1**) ∈ ℝ^*K*×*K*^ is the diagonal matrix.

#### 3.3.2. Spectral Analysis on Global Fused Similarity Matrix

To further simplify the clustering process, spectral clustering can be performed on the global fused similarity matrix **S**. Specifically, the objective function of spectral clustering is

(8) $$\begin{array}{c} \underset{F^{T}F=I}{\min}\text{tr}\left(F^{T}LF\right), \end{array}$$

where tr(·) is the matrix trace operator, **F** ∈ ℝ^*N*×*K*^ is the indicator matrix, and *K* is the number of clusters. The Laplacian matrix **L** is defined as **L** = **D** − **S** in graph theory, where the degree matrix **D** ∈ ℝ^*N*×*N*^ is written as a diagonal matrix with **D**_*ii*_ = ∑_*j*=1_^*N*^**S**_*ij*_. We can obtain the indicator matrix **F** that consists of eigenvectors corresponding to the largest *K* eigenvalues by performing eigen decomposition on **L**. However, the computational complexity is *𝒪*(*N*^2^*K*) via performing eigen decomposition on **L**, which leads to being not suitable for large-scale data.

Fortunately, according to [2, 37], **S** is a double stochastic matrix. Thus, the degree matrix **D** = diag(**S1**) is an identity matrix **I**, and the Laplacian matrix **L** can be written as **L** = **I** − **S**. To make the analysis simple, (8) is equivalent to the following equation:

(9) $$\begin{array}{c} \underset{F^{T}F=I}{\max}\text{tr}\left(F^{T}SF\right). \end{array}$$

Note that **S** can be written as **S** = **ZΛ**^−1^**Z**^*T*^ = **ZΛ**^−1/2^**Λ**^−1/2^**Z**^*T*^ = **AA**^**T**^, where **A** = **ZΛ**^−1/2^ and **A** ∈ ℝ^*N*×*K*^. The Singular Value Decomposition (SVD) of **A** can be formulated as

(10) $$\begin{array}{c} A=U\Sigma V^{T}, \end{array}$$

where **U** ∈ ℝ^*N*×*N*^, **Σ** ∈ ℝ^*N*×*K*^, and **V** ∈ ℝ^*K*×*K*^ are the left singular vector matrix, singular value matrix, and right singular vector matrix, respectively. Furthermore, **U** and **V** satisfy both **U**^*T*^**U** = **I** and **V**^*T*^**V** = **I**. Thus **S** can be derived from (10) as

(11) $$\begin{array}{c} S=AA^{T}=\left(U\Sigma V^{T}\right){\left(U\Sigma V^{T}\right)}^{T}=U\left(\Sigma \Sigma^{T}\right)U^{T}. \end{array}$$

It is obvious that the column vectors of **U** are the eigenvectors of the similarity matrix **S**. To reduce the computational complexity, we prefer to conduct SVD on **A** to acquire the desired **F** rather than to directly perform eigenvalue decomposition on **S**. Based on this, (10) is written as

(12) $$\begin{array}{c} U=AV\Sigma^{-1}. \end{array}$$

Since **Σ** and **V** are the singular value matrix and right singular vector matrix of **A**, respectively, we can perform eigen decomposition on a small *K* × *K* matrix **R** = **A**^*T*^**A** = **Λ**^−1/2^**Z**^*T*^**ZΛ**^−1/2^, resulting in *K* eigenvector-eigenvalue pairs {(**v**_*i*_, **θ**_*i*_)}_*i*=1_^*K*^, where 1 > **θ**_1_ ≥ …≥**θ**_*K*_ > 0. We denote by **V** = [**v**_1_,…, **v**_*K*_] ∈ ℝ^*K*×*K*^ a column-orthonormal matrix containing the *K* eigen vectors and by Θ = diag(**θ**_1_,…, **θ**_*K*_) ∈ ℝ^*K*×*K*^ a diagonal matrix storing the *K* eigen values on the main diagonal. It is obvious that

(13) $$\begin{array}{c} R=A^{T}A={\left(U\Sigma V^{T}\right)}^{T}\left(U\Sigma V^{T}\right)=V\left(\Sigma^{T}\Sigma \right)V^{T}, \end{array}$$

where **Σ**^*T*^**Σ** returns a *K* × *K* diagonal matrix storing all the eigen values of **R** = **A**^*T*^**A**. Thus, the singular value matrix **Σ** can be derived as **Σ** = Θ^1/2^. Then, the final solution can be simplified as

(14) $$\begin{array}{c} F=Z\Lambda^{-1/2}V\Theta^{-1/2}, \end{array}$$

where **F** ∈ ℝ^*N*×*K*^ is the indicator matrix. After that, we can perform semi-supervised *K*-Means on **F** to acquire the final results. The whole procedure of SMVC_WAGE for complete multi-view data is summarized in Algorithm 1.

### 3.4. The Proposed Method for Incomplete Multi-View Data

Our proposed method (SMVC_WAGE) can not only deal with complete multi-view clustering well, but also be easily extended to incomplete multi-view clustering. To simplify the incomplete multi-view case, we take three views as an example, which verifies that SMVC_WAGE can be straightforwardly extended to the scenarios of incomplete multi-view data.

Similar to the problem definition in Section 3.1, we still assume that the incomplete three-view data consists of *N* samples. In order to make the discussion easy without losing generality, we follow [2] to adjust the original dataset to *𝒳* = {**X**^(1,2,3)^, **X**^(1,2)^, **X**^(1,3)^, **X**^(2,3)^, **X**^(1)^, **X**^(2)^, **X**^(3)^}, where **X**^(1,2,3)^ ∈ ℝ^*n*_*c*_×(*d*_1_ + *d*_2_ + *d*_3_)^, **X**^(1,2)^ ∈ ℝ^*n*_12_×(*d*_1_ + *d*_2_)^, **X**^(1,3)^ ∈ ℝ^*n*_13_×(*d*_1_ + *d*_3_)^, **X**^(2,3)^ ∈ ℝ^*n*_23_×(*d*_2_ + *d*_3_)^, **X**^(1)^ ∈ ℝ^*n*_1_×*d*_1_^, **X**^(2)^ ∈ ℝ^*n*_2_×*d*_2_^, and **X**^(3)^ ∈ ℝ^*n*_3_×*d*_3_^ denote the samples present in the three views, both view-1 and view-2, both view-1 and view-3, both view-2 and view-3, only view-1, only view-2, and only view-3, respectively. Similarly, *n*_*c*_ is the number of samples described by the three views. *n*_12_ denotes the number of samples shared by both view-1 and view-2; *n*_13_ and *n*_23_ have the same meaning. *n*_*v*_(*v* = 1,2,3) stands for the number of samples only existing in the *v*-th view. The total number of samples is *N* = *n*_*c*_ + *n*_12_ + *n*_13_ + *n*_23_ + *n*_1_ + *n*_2_ + *n*_3_.

As stated in Section 3.3, the proposed method (SMVC_WAGE) for incomplete multi-view data mainly consists of two steps, i.e., construction of anchor-based global fused similarity matrix **S** and spectral analysis of a global fused similarity matrix.  Figure 1 shows the whole construction process of the global fused similarity matrix, and all possible cases are considered in incomplete three-view data, i.e., missing two views, missing one view, and missing no view.

It is very challenging to randomly choose from labeled data to generate anchor points in incomplete multi-view data, as some labeled samples miss one view or two views, and thus pairwise information may be unavailable. Fortunately, the common samples appearing in all views can help generate anchor points to solve the dilemma. Based on the above analysis, we assume that all labeled samples covering each cluster are included in common samples; then, we can obtain the seed set ${𝒳}_{𝒮}=\left\{X_{S}^{\left(1,2,3\right)},\hat{y}\right\}$ from the common samples with the label, where **X**_*S*_^(1,2,3)^ ∈ ℝ^*q*×(*d*_1_ + *d*_2_ + *d*_3_)^ denotes the seed set present in all views, $\hat{y}=\left[{\hat{y}}_{1};{\hat{y}}_{2};\ldots ;{\hat{y}}_{q}\right]\in {\mathbb{R}}^{q}$ denotes the corresponding label vector, and *q* represents the number of samples in the seed set. Then, as stated in Section 3.3.1, the generated anchor points set in the *v*-th view can be represented as **U**^(*v*)^ = [**u**_1_^(*v*)^; **u**_2_^(*v*)^; …; **u**_*K*_^(*v*)^] ∈ ℝ^*K*×*d*_*v*_^, where **u**_*l*_^(*v*)^ can be obtained according to (2).

As illustrated in the second column in Figure 1, we partition this incomplete three-view case into three scenarios. Specifically, we rearrange the samples according to the characteristics of each sample so that we can directly perform the anchor-based truncated similarity matrix construction method described in Section 3.3.1 on each scenario. Each scenario can be represented as a view and the view's anchor points, where missing samples are removed. Taking the first scenario as an example, there are *n*_*c*_ + *n*_12_ + *n*_13_ + *n*_1_ samples that appeared in view-1, and *n*_*k*_ anchor points are generated from the seed set **X**_*S*_^(1,2,3)^. Then, we construct an anchor-based truncated similarity matrix **Z**^(1)^ ∈ ℝ^(*n*_*c*_ + *n*_12_ + *n*_13_ + *n*_1_)×*n*_*k*_^ by (4). Similarly, we can analyze other scenarios.

To fuse the above truncated similarity matrices that appeared in three scenarios appropriately, we reorder them into aligned matrices, with rows and columns following the order of the original samples. To fully exploit the consistent and complementary information among different views, we make the view with high quality have a larger weight ratio in the common representation by employing the prior knowledge from multi-view data. More specifically, we first obtain the clustering accuracy **a**_*v*_ of each view in the seed set ${𝒳}_{𝒮}=\left\{X_{S}^{\left(1,2,3\right)},\hat{y}\right\}$ and apply softmax function to acquire the weight **w** for different views as mentioned in Section 3.3.1. Then, we obtain the global truncated similarity matrix **Z** ∈ ℝ^*N*×*n*_*k*_^ according to the weighted combining scheme by (6). Finally, we acquire the global fused similarity matrix **S** ∈ ℝ^*N*×*N*^ by (7) as Figure 1 shows.

According to Section 3.3.2, as a final step, spectral clustering is performed on the global fused similarity matrix **S** to acquire a unified clustering result. The whole procedure of SMVC_WAGE for incomplete three-view data is summarized in Algorithm 2.

### 3.5. Theoretical Analysis of the Proposed Algorithm

In this section, we provide a brief theoretical analysis of the proposed algorithm, containing computational complexity analysis and convergence analysis.

#### 3.5.1. Computational Complexity Analysis

The computational complexity of the proposed algorithm mainly consists of five parts, i.e., calculating **U**^(*v*)^, **Z**^(*v*)^, **w**_*v*_, **F**, and the final clustering results. In Algorithm 1, the corresponding computation is in steps 3, 4, 6, 9, and 10, where the number of anchor points and clusters, expressed in *K*, is equal for each view. Specifically, computation complexity of these steps is summarized as follows:

1. Obtaining anchor points set **U**^(*v*)^ containing *K* anchor points requires *𝒪*(1)
2. Obtaining the truncated similarity matrix **Z**^(*v*)^ requires *𝒪*(*NKd*_*v*_) according to (4)
3. Obtaining the weight **w**_*v*_ requires *𝒪*(*t*_*v*_*qKd*_*v*_) + *𝒪*(*K*^2^) according to (5) and (17), where *t*_*v*_ and *q* are the iterative number and the number of labeled samples, respectively, when performing semi-supervised *K*-Means for each view
4. Obtaining the indicator matrix **F** requires *𝒪*(*K*^3^) by performing eigen decomposition on **R** = **A**^*T*^**A** according to (13)
5. Obtaining the final clustering results requires *𝒪*(*tNK*^2^) by performing semi-supervised *K*-Means, where *t* is the iterative number

Therefore, the total main computational complexity of Algorithm 1 is

(15) $$\begin{array}{c} O\left(\sum_{v=1}^{V}\left(1+NKd_{v}+t_{v}qKd_{v}+K^{2}\right)+K^{3}+tNK^{2}\right). \end{array}$$

Note that the dataset's view number *V* ≪ *N*, clusters or anchor points number *K* ≪ *d* and *K* ≪ *N*, and the number of labeled samples *q* depends on the samples number *N* and the percentage of labeled data *ξ*. Since we exploit semi-supervised *K*-Means to obtain the clustering result, *t*_*v*_ and *t* are usually small [38].

Compared with Algorithm 1, the main difference of Algorithm 2 is to deal with incomplete multi-view data. Therefore, similar to the Algorithm 1, the total main computational complexity of Algorithm 2 is

(16) $$\begin{array}{c} O\left(\sum_{v=1}^{V}\left(1+N_{v}Kd_{v}+t_{v}qKd_{v}+K^{2}\right)+K^{3}+tNK^{2}\right), \end{array}$$

where *N*_*v*_ denotes the number of non-missing samples in the *v*-th view.

According to the above analysis, in order to further simplify the representation, the overall computational complexity of SMVC_WAGE is *𝒪*(*Nd* + *qd* + *N*), where *d* = max(*d*_1_, *d*_2_,…, *d*_*V*_). In addition, the experimental results of running time have also proven the computational advantages of SMVC_WAGE.

#### 3.5.2. Convergence Analysis

Firstly, the whole procedure of SMVC_WAGE just exploits the semi-supervised *K*-Means to calculate the optimal clustering result in an iterative manner, where the strong convergence property of semi-supervised *K*-Means has been proven in [38, 39]. Secondly, by calculating (13) performing eigen decomposition, indicator matrix **F** can obtain the global optimal solution [9]. Thirdly, the experimental result of convergence study can also demonstrate the strong convergence of SMVC_WAGE. In summary, the proposed method has good convergence property.

## 4. Experiments

In this section, extensive experiments are performed to evaluate the performance of our method (SMVC_WAGE). Firstly, we describe six multi-view datasets used in the experiment. Secondly, we introduce the comparative methods and evaluation metrics. Ultimately, the comparison results show the proposed method's effectiveness and efficiency.

### 4.1. Datasets Description

Six real-world multi-view datasets are adopted to validate our method. Among these datasets, the first two are text datasets, and the other four are image datasets. They are widely used benchmark datasets. The descriptions of these datasets are given below, and some important statistical information is presented in Table 1.

1. Cornell (http://lig-membres.imag.fr/grimal/data.html): this text dataset is one of the popular WebKB datasets [3, 26]. It includes 195 documents with more than 5 labels: student, project, course, staff, and faculty, where each document is characterized by two views: the citation view and the content view, i.e., 195 citation features and 1703 content features.
2. 3Sources (http://erdos.ucd.ie/datasets/3sources.html): this text dataset is naturally an incomplete multi-view dataset [2] and is collected from three well-known online news sources: BBC, Reuters, and The Guardian. In total, it contains 948 news articles covering 416 distinct news stories, which are categorized into six topical labels: business, entertainment, health, politics, sport, and technology. Among these distinct stories, 53 appear in a single news source, 194 are in two sources, and 169 are reported in all three sources.
3. UCI Handwritten Digit (http://archive.ics.uci.edu/ml/datasets/Multiple+Features): this image dataset consists of 2000 samples of hand-written numerals (0–9) extracted from Dutch utility maps. Each class has 200 samples. There are six different types of features which can be used for performing multi-view learning, that is, 76 Fourier coefficients of the character shapes, 216 profile correlations, 64 Karhunen–Loève coefficients, 240 pixel averages in 2 × 3 windows, 47 Zernike moments, and 6 morphological features [31].
4. ORL (http://www.cad.zju.edu.cn/home/dengcai/Data/FaceData.html): this image dataset contains 400 images of 40 distinct individuals with 10 different images which were taken at different times, varying the lighting, facial expressions, and facial details [40]. Following experiments in [41], we used three feature sets: 4096 dimension intensity feature, 3304 dimension LBP feature, and 6750 dimension Gabor feature.
5. NUS-WIDE-OBJECT (NUS) (https://lms.comp.nus.edu.sg/wp-content/uploads/2019/research/nuswide/NUS-WIDE.html): this image dataset is a real-world web image dataset. There are 31 object categories and 30000 images in total [42]. In our experiments, 7 categories of the animal concept are selected. They are bear, cow, elk, fox, horses, tiger, and zebra. Each image can be represented by five public available low-level features on its homepage website: 64 dimension color histogram (CH), 225 dimension color moments (CM), 144 dimension color correlation (CORR), 73 dimension edge distribution (ED), and 128 wavelet texture (WT).
6. MSRC-v1 (https://www.microsoft.com/en-us/research/project/image-understanding/): this image dataset contains 240 images in eight categories, and each category has 30 images [43]. Following experiments in [29], we select seven categories: tree, building, airplane, cow, face, car, and bicycle. Each image is represented by five features: 24 dimension Color Moment (CM), 576 dimension Histogram of Oriented Gradient (HOG), 512 dimension GIST, 256 dimension Local Binary Pattern (LBP), and 254 Centrist features (CENTRIST).

### 4.2. Compared Methods and Experimental Settings

Our proposed method solves the problem of complete and incomplete multi-view clustering. Thus, to prove the efficiency and effectiveness of this framework, we choose Spectral Clustering [44] and three multi-view methods to compare the performance of complete multi-view clustering: MVSC [6], AMGL [29], and MLAN [45]. Similarly, we compare the Spectral Clustering [44], PVC [21], IMG [22], DAIMC [24], IMSC_AGL [26], and APMC [2] for incomplete multi-view clustering. We denote the proposed method as SMVC_WAGE. The description of these methods is given as follows:

1. SC: we perform Spectral Clustering (SC) [44] on all views independently as the baseline.
2. SC (concat): we firstly concatenate all views into long dimension features and then run Spectral Clustering [44] to acquire the result.
3. MVSC: Multi-View Spectral Clustering (MVSC) [6] constructs a bipartite graph and then uses local manifold fusion to integrate the graph of each view into a fused graph. Finally, Spectral Clustering is performed on the fused graph to obtain the result.
4. AMGL: Auto-weighted Multiple Graph Learning (AMGL) [29] is a Spectral Clustering-based method and is easily extended to semi-supervised multi-view clustering. It automatically learns a set of optimal weights without any parameters.
5. MLAN: Multi-view Learning with Adaptive Neighbors (MLAN) [45] is a graph-based multi-view learning model and calculates the ideal weights automatically after finite iterations. It can perform local manifold structure learning and semi-supervised clustering simultaneously.
6. PVC: Partial multi-View Clustering (PVC) [21] works based on non-negative matrix factorization to acquire a consistent representation. Lastly, *K*-Means is performed on the consistent representation to acquire the result.
7. IMG: Incomplete Multi-modal Grouping (IMG) [22] utilizes matrix factorization techniques to obtain the consistent representation. It learns the compact global structure from the latent consistent representation, and lastly *K*-Means is performed on the consistent representation to acquire the result.
8. DAIMC: Doubly Aligned Incomplete Multi-view Clustering (DAIMC) algorithm [24] learns a latent consistent representation from all views via integrating weighted semi-NMF and *L*_2,1_-norm regularized regression. Lastly, *K*-Means is performed on the latent consistent representation to acquire the result.
9. IMSC_AGL: Incomplete Multi-view Spectral Clustering with Adaptive Graph Learning (IMSC_AGL) [26] integrates the spectral clustering and adaptive graph learning technique to obtain the latent consistent representation from all views. Lastly, it partitions the samples into their respective groups via *K*-Means clustering.
10. APMC: Anchor-based Partial Multi-view Clustering (APMC) [2] utilizes anchors to integrate intra- and inter-view similarity matrices, and then Spectral Clustering is performed on the fused similarity matrix to acquire the unified result.

For comparison methods, the source codes are available from the authors' websites. Since the 3Sources dataset is a naturally incomplete multi-view dataset, we utilize it for incomplete multi-view clustering and conduct complete multi-view clustering on the other datasets. We select the best two views from the 3Sources dataset as the input of PVC and IMG, because they cannot work on more than two-view scenario. Since SC cannot directly deal with incomplete multi-view data, we first populate the missing information with the mean of the feature values in the corresponding view. Empirically, the number of nearest neighbors accounts for 10% of the dataset size. Since all the comparison methods conduct *K*-Means clustering on the latent consistent representation, we set the maximum number of iterations to 1000 for *K*-Means clustering. Considering the limitation of the comparison methods, we firstly learn a latent consistent representation of the raw data and then use labeled data to generate seed clusters that are utilized to initialize the cluster centroids of semi-supervised *K*-Means. Furthermore, to make the experiments more conclusive and fair, the parameters of each method are initialized, being corresponding to the paper's report, and present the final result of SMVC_WAGE with the trade-off parameter *λ* = 10 and the width parameter *σ* = 1 in Gaussian kernel function. In terms of semi-supervised clustering, for all datasets, we randomly choose a small proportion as labeled data in each category, where the proportion is denoted by *ξ*(10%, 20%, 30%, 40%). To randomize the experiment, we run each method 20 times with different random initialization to record the mean performance as well as the standard deviations in all experiments. Due to different parameter ranges and preprocessing, some of the results may be inconsistent with the published information.

### 4.3. Evaluation Metrics

There are many evaluation metrics for assessing the clustering performance [46]. In our experiments, we choose three evaluation metrics, namely, Clustering Accuracy (ACC), Normalized Mutual Information (NMI), and Purity, to conduct a comprehensive evaluation. These evaluation metrics can be calculated in a certain framework through the clustering result and the ground-truth of the dataset.

The first evaluation metric is ACC, usually defined as follows:

(17) $$\begin{array}{c} \text{ACC}=\frac{\sum_{i=1}^{n}\delta \left(\text{map}\left(c_{i}\right),y_{i}\right)}{n}, \end{array}$$

where *n* means the number of samples, *y*_*i*_ means the ground-truth label of the *i*-th sample, *c*_*i*_ means the corresponding cluster label calculated, *δ* means the Dirac delta function:

(18) $$\begin{array}{c} \delta \left(x,y\right)=\left\{\begin{array}{cc} 1, & \text{if }x=y,\\ 0, & \text{otherwise,} \end{array}\right. \end{array}$$

and map(·) is the optimal mapping function that arranges the cluster labels to match the ground-truth labels via the Kuhn–Munkres algorithm [47].

The second evaluation metric is NMI, which integrates mutual information and entropy. NMI is formulated as follows:

(19) $$\begin{array}{c} \text{NMI}\left(c_{i},y_{i}\right)=\frac{I\left(c_{i},y_{i}\right)}{\sqrt{E\left(c_{i}\right)E\left(y_{i}\right)}}, \end{array}$$

where *I*(*y*_*i*_, *c*_*i*_) denotes the mutual information between *y*_*i*_ and *c*_*i*_, and *E*(·) returns the entropy.

Let *n*_*i*_^*c*^ be the number of samples in cluster *C*_*i*_(1 ≤ *i* ≤ *k*) which is acquired via performing clustering methods, and *n*_*j*_^*y*^ be the number of samples belonging to cluster *Y*_*j*_(1 ≤ *j* ≤ *k*) with the ground-truth label. Then, NMI is rewritten as

(20) $$\begin{array}{c} \text{NMI}=\frac{\sum_{i=1}^{k}\sum_{j=1}^{k}n_{i,j}\log\left(n\cdot n_{i,j}/n_{i}^{c}\cdot n_{j}^{y}\right)}{\sqrt{\left(\sum_{i=1}^{k}n_{i}^{c}\log\left(n_{i}^{c}/n\right)\right)\left(\sum_{j=1}^{k}n_{j}^{y}\log\left(n_{j}^{y}/n\right)\right)}}, \end{array}$$

where *n*_*i*,*j*_ means the number of samples in the intersection between *C*_*i*_ and *Y*_*j*_.

The third evaluation metric is Purity which measures the effectiveness of clustering by calculating the percentage of correct labels. Purity is defined by

(21) $$\begin{array}{c} \text{Purity}=\frac{1}{n}\sum_{i=1}^{k}\underset{1\leq j\leq k}{\max}\left|C_{i}\cap Y_{j}\right|. \end{array}$$

For the three evaluation metrics, a higher value indicates a better performance. The readers can refer to [48] to get more details about their definitions.

### 4.4. Experimental Results and Analysis

#### 4.4.1. Complete Multi-View Clustering Results

To explore the effectiveness of our method, these complete multi-view methods are performed on five complete multi-view datasets with different percentages of labeled data, where the experimental results are enumerated in Tables 2–6 in the form of ACC, NMI, and Purity. Through the analysis of these tables, we can get some observations as follows:

1. From Tables 2–6, we can see that the clustering performances are quite different in single-view clustering scenarios for all multi-view datasets. This is mainly because each view has a difference in the feature scales and distributions. The experimental results also imply that it is necessary to research how to appropriately combine multiple views to enhance the clustering performance.
2. From Tables 2–6 and Figures 2(a)–2(e), we can find that the proposed SMVC_WAGE can obtain much better results than the best single view and concat for all scenarios. Meanwhile, we can see that concat performs the worst in most instances, mainly because directly concatenating views into a long view may lead to redundant information, resulting in poor clustering results. Thus, these experiment results demonstrate that clustering performance can be effectively improved via properly exploiting the consistent and complementary information to learn a common representation.
3. From Tables 2–6, we can see that the proposed SMVC_WAGE outperforms all competitors such as MVSC, AMGL, and MLAN while dealing with most of the complete multi-view clustering. This is mainly because SMVC_WAGE can not only fully exploit the intrinsic consistency and extrinsic complementary information across different views, but also make the high-quality single view has a larger weight ratio in the common representation by utilizing the prior information in the multi-view data. These experimental results prove that our method is effective in complete multi-view clustering.
4. From Tables 2–6, we observe that the performance of the above methods first rises to high value and then maintain slight variation as the number of labeled data increases. For the proposed SMVC_WAGE, with 30% or 40% labeled data, the method always obtains the best result. Meanwhile, with 10% or 20% labeled data, our method obtains slightly worse results. The main reason is that our method heavily depends on how to construct the graph through prior information. Thus, we cannot generate the structure of the graph optimally when there is less labeled data, leading to slightly worse results.

#### 4.4.2. Incomplete Multi-View Clustering Results

To explore the effectiveness of the presented SMVC_WAGE in dealing with the incomplete multi-view data, we conduct experiments on the naturally incomplete 3Sources dataset, where the missing rate of each view is 16%, 28%, and 30%, respectively. The results are recorded in Table 7 and Figure 2(f). Similar to the complete multi-view clustering, the above comparison results show that the performance of the proposed SMVC_WAGE is significantly superior to all the compared methods on the 3Sources dataset with a different percent of labeled data. Thus, our method can deal with incomplete multi-view clustering well.

The above experimental results on Cornell, UCI Handwritten Digit, ORL, NUS-WIDE-OBJECT, MSRC-v1, and 3Sources have well proven that the presented SMVC_WAGE outperforms most algorithms in terms of clustering ability. The main reason is that SMVC_WAGE firstly introduces an effective and simple anchor strategy that can bridge all samples and capture more reliable nonlinear relations to deal with both complete and incomplete multi-view data. Besides, it exploits the intrinsic consistency and extrinsic complementary information to learn a structured optimal fused graph in a semi-supervised clustering weighting manner, which can greatly enhance efficiency and improve stableness.

### 4.5. Running Time

The running time was recorded to compare the computational complexity of the methods on all datasets. From Table 8, it is clear that the proposed SMVC_WAGE has the shortest running time in almost all datasets except MSRC-v1. Meanwhile, as shown in Figure 3, in which the original data is from Table 8, we see that the running time of SMVC_WAGE is many times smaller than the above-mentioned multi-view clustering algorithms on all datasets, especially the UCI Handwritten Digit, ORL, NUS-WIDE-OBJECT, and 3Sources dataset. This is mainly because these datasets have a relatively large number of views and samples, and the data quality of each view varies greatly. In summary, the experimental results have fully proven the computational advantages of SMVC_WAGE.

### 4.6. Parameter Sensitivity Analysis

Our proposed SMVC_WAGE has only one hyperparameter *λ*, which trades off the weight of each view. In the following, the parameter analytical experiments are performed on each dataset to reveal the effect of this parameter. We first set the percentage of labeled data *ξ* from 10% to 40% as mentioned before; then, we explore the ACC of SMVC_WAGE by ranging the *λ* within {0.01, 0.1, 1,10,100} and record the average performances. As shown in Figures 4(a) and 4(d), we observe that, with *λ* increasing from 0.01 to 100, the mean of ACC with fixed *ξ* first increases to high value and then decreases. Regarding Figures 4(b)–4(f), similarly, we observe that the result of SMVC_WAGE increases first and then maintains slight variation. Therefore, SMVC_WAGE can obtain a stable great performance across a wide range of *λ*. Obviously, the performance keeps optimal in *λ* = 10. These experiments have fully demonstrated that SMVC_WAGE is not so sensitive to the variation of the hyperparameter *λ* in the final results.

### 4.7. Convergence Study

To investigate the convergence empirically, we record ACC of SMVC_WAGE in every iteration on each dataset where we set the percentage of labeled data *ξ* = 10% and the hyperparameter *λ* = 10, respectively. For a full iteration, SMVC_WAGE firstly calculates the clustering accuracy for all views via performing semi-supervised *K*-Means in order to obtain the global fused similarity matrix. In this process, the final ACC is not calculated, but it will consume some time. Without loss of generality, we will use semi-supervised *K*-Means as an iteration each time, while recording the final ACC. We plot ACC in Figure 5. For each subfigure, we can see that the value of the ACC is zero in the first multiple iterations at the beginning because our algorithm uses the prior information of the data, and after a finite number of iterations, the ACC begins to increase and gradually stabilize. Moreover, it reveals that SMVC_WAGE usually converges within 50 iterations for all datasets, which empirically proves the high efficiency of our algorithm.

## 5. Conclusion

In this paper, a new semi-supervised multi-view clustering framework is developed, which is conceptually simple and efficiently generates high-quality clustering results in practice. Specifically, our method introduces a simple and effective anchor strategy that exploits the intrinsic and extrinsic view information to bridge all samples and capture more reliable nonlinear relations, which can greatly enhance efficiency and improve stableness. Besides, this can also solve the dilemma that samples sharing no common views cannot be directly used for computing cross-view similarities. Meanwhile, instead of regularizing or weighting the loss of each view in a conventional way, the proposed method constructs the global fused graph that spans multiple views compatibly in the structure via a parameter-free graph fusion mechanism which directly coalesces the view-wise graphs. To this end, the proposed method can not only deal with complete multi-view clustering well, but also be easily extended to the incomplete multi-view instance. Experimental results on six widely used real-world datasets clearly show that our proposed algorithm is superior to some state-of-the-art competitors in clustering ability and time cost.

When handling incomplete multi-view clustering, we found that the main limitation of this approach may be that anchor points can only be generated from common samples appearing in all views, which remains to be further studied.

## Figures and Tables

**Figure 1:** Anchor-based global fused similarity matrix construction for incomplete three-view data.

**Figure 2:** ACC (%) of SMVC_WAGE, SC (the best single view), and SC (concat) on six real-world datasets with a different percent of labeled data: (a) Cornell; (b) UCI Handwritten Digit; (c) ORL; (d) NUS-WIDE-OBJECT; (e) MSRC-v1; (f) 3Sources.

**Figure 3:** The average running time (seconds) of methods mentioned above on each dataset. In the figure, to ensure visual discernibility, the running time of maximum display is 5 seconds in the coordinate axis, and the specific value can be seen in Table 8: (a) the five complete datasets: Cornell, Digit, ORL, NUS, and MSRC-V1; (b) the incomplete dataset: 3Sources dataset.

**Figure 4:** The performance of SMVC_WAGE in a different value of the parameter *λ* and *ξ*: (a) Cornell; (b) UCI Handwritten Digit; (c) ORL; (d) NUS-WIDE-OBJECT; (e) MSRC-v1; (f) 3Sources.

**Figure 5:** The value of ACC (%) in different iterative steps is acquired via running SMVC_WAGE on six datasets with *λ* = 10 and *ξ* = 10%: (a) Cornell; (b) UCI Handwritten Digit; (c) ORL; (d) NUS-WIDE-OBJECT; (e) MSRC-v1; (f) 3Sources.

**Algorithm 1:** The proposed SMVC_WAGE for complete multi-view data.

**Algorithm 2:** The proposed SMVC_WAGE for incomplete three-view data.

**Table 1:** Statistics of multi-view datasets used in our experiments.

Dataset	# samples	# clusters	# views	# features
Cornell	195	5	2	1703/195
3Sources	416	6	3	3560/3631/3068
Digit	2000	10	6	76/216/64/240/47/6
ORL	400	40	3	4096/3304/6750
NUS	2833	7	5	64/225/144/73/128
MSRC-v1	210	7	5	24/576/512/256/254

**Table 2:** Aggregated ACC (%), NMI (%), and Purity (%) comparison (mean ± std) of different methods on Cornell dataset with a different percent of labeled data.

*ξ*	10%			20%			30%			40%		
	ACC	NMI	Purity	ACC	NMI	Purity	ACC	NMI	Purity	ACC	NMI	Purity
SC (1)	33.41 ± 3.61	7.14 ± 2.18	44.74 ± 1.90	31.97 ± 2.25	6.56 ± 1.96	44.00 ± 1.64	32.56 ± 3.25	6.92 ± 2.38	44.41 ± 2.01	32.64 ± 2.68	7.43 ± 1.67	44.77 ± 1.37
SC (2)	41.64 ± 1.22	19.84 ± 1.52	57.36 ± 2.36	41.28 ± 0.95	19.63 ± 1.26	57.44 ± 1.32	41.00 ± 0.72	19.34 ± 1.29	56.87 ± 1.19	41.13 ± 1.16	18.89 ± 1.62	56.67 ± 1.71
SC (concat)	34.31 ± 2.30	10.46 ± 1.84	46.56 ± 2.17	34.31 ± 1.69	9.97 ± 1.58	46.00 ± 1.96	35.23 ± 2.02	10.49 ± 2.23	47.44 ± 1.83	35.21 ± 1.85	9.94 ± 1.42	47.49 ± 1.49
MVSC	32.92 ± 2.35	3.61 ± 1.49	43.23 ± 0.73	32.49 ± 0.88	5.59 ± 1.13	46.15 ± 1.20	33.95 ± 0.54	7.75 ± 0.48	44.08 ± 0.39	34.15 ± 1.67	5.78 ± 0.46	44.23 ± 0.60
AMGL	39.23 ± 4.43	15.37 ± 1.85	50.21 ± 2.70	38.05 ± 3.21	15.14 ± 1.99	49.18 ± 2.88	39.59 ± 2.80	16.32 ± 1.61	50.13 ± 1.49	38.56 ± 2.40	15.71 ± 1.79	49.38 ± 2.31
MLAN	43.10 ± 2.41	24.89 ± 0.70	55.38 ± 0.00	43.15 ± 2.64	24.89 ± 0.67	55.38 ± 0.00	42.21 ± 1.61	24.78 ± 1.19	55.28 ± 0.46	42.56 ± 0.00	25.04 ± 0.00	55.38 ± 0.00
SMVC_WAGE	**63.49** ± **6.95**	**37.11** ± **7.17**	**66.31** ± **5.56**	**73.90** ± **3.36**	**51.67** ± **3.95**	**75.67** ± **2.41**	**78.08** ± **1.86**	**55.32** ± **2.73**	**78.18** ± **1.82**	**81.36** ± **3.36**	**61.28** ± **5.18**	**81.51** ± **3.19**

Bold numbers denote the best results.

**Table 3:** Aggregated ACC (%), NMI (%), and Purity (%) comparison (mean ± std) of different methods on UCI Handwritten Digit dataset with a different percent of labeled data.

*ξ*	10%			20%			30%			40%		
	ACC	NMI	Purity	ACC	NMI	Purity	ACC	NMI	Purity	ACC	NMI	Purity
SC (1)	21.04** **±** **2.75	9.24 ± 3.65	22.32 ± 3.03	20.65 ± 2.01	8.70 ± 2.91	21.94 ± 2.33	20.94 ± 2.60	9.46 ± 2.93	22.06 ± 2.54	20.88 ± 2.46	9.65 ± 3.92	22.15 ± 2.85
SC (2)	66.77** **±** **0.43	59.46 ± 0.66	66.77 ± 0.43	66.60 ± 0.66	59.28 ± 0.84	66.61 ± 0.63	66.65 ± 0.56	59.32 ± 0.74	66.67 ± 0.52	66.70 ± 0.38	59.42 ± 0.53	66.70 ± 0.38
SC (3)	18.00** **±** **1.19	6.73 ± 1.36	19.96 ± 1.53	18.63 ± 1.04	7.17 ± 1.08	20.24 ± 1.24	18.12 ± 1.08	6.64 ± 1.21	19.78 ± 1.16	17.63 ± 1.08	6.23 ± 0.90	19.18 ± 0.98
SC (4)	55.82** **±** **1.36	46.79 ± 1.12	55.89 ± 1.46	55.80 ± 1.46	46.68 ± 1.08	55.84 ± 1.51	55.55 ± 1.04	46.53 ± 0.89	55.60 ± 1.15	55.27 ± 1.01	46.26 ± 0.72	55.27 ± 1.01
SC (5)	75.41** **±** **0.02	68.49 ± 0.05	75.41 ± 0.02	75.41 ± 0.02	68.50 ± 0.06	75.41 ± 0.02	75.40 ± 0.01	68.48 ± 0.04	75.40 ± 0.01	75.40 ± 0.02	68.49 ± 0.05	75.40 ± 0.02
SC (6)	43.54** **±** **0.91	38.45 ± 0.50	44.28 ± 0.57	43.91 ± 0.51	38.51 ± 0.38	44.43 ± 0.56	44.34 ± 0.56	38.67 ± 0.32	44.91 ± 0.64	44.12 ± 0.61	38.44 ± 0.56	44.61 ± 0.72
SC (concat)	79.00 ± 0.05	73.48 ± 0.12	79.00 ± 0.05	78.98 ± 0.04	73.44 ± 0.11	78.98 ± 0.04	78.98 ± 0.04	73.44 ± 0.11	78.98 ± 0.04	78.96 ± 0.03	73.40 ± 0.08	78.96 ± 0.03
MVSC	50.11 ± 1.92	42.80 ± 0.97	54.12 ± 1.52	50.05 ± 2.16	43.43 ± 1.82	54.09 ± 2.53	51.44 ± 2.31	43.78 ± 1.38	55.09 ± 2.04	51.06 ± 1.16	44.11 ± 0.72	55.00 ± 0.94
AMGL	88.40** **±** **0.00	89.11** **±** **0.00	88.40** **±** **0.00	88.40** **±** **0.00	89.11** **±** **0.00	88.40** **±** **0.00	88.40** **±** **0.00	89.11** **±** **0.00	88.40** **±** **0.00	88.40** **±** **0.00	89.11** **±** **0.00	88.40** **±** **0.00
MLAN	**97.30 **±** 0.00**	**93.91 **±** 0.00**	**97.30 **±** 0.00**	**97.30 **±** 0.00**	**93.91 **±** 0.00**	**97.30 **±** 0.00**	**97.30 **±** 0.00**	**93.91 **±** 0.00**	**97.30 **±** 0.00**	**97.35 **±** 0.00**	**94.00 **±** 0.00**	**97.35 **±** 0.00**
SMVC_WAGE	91.33 ± 0.83	82.98 ± 1.25	91.33 ± 0.83	91.69 ± 0.44	83.60 ± 0.73	91.69 ± 0.44	91.98 ± 0.27	84.00 ± 0.52	91.98 ± 0.27	92.24 ± 0.33	84.42 ± 0.64	92.24 ± 0.33

Bold numbers denote the best results.

**Table 4:** Aggregated ACC (%), NMI (%), and Purity (%) comparison (mean ± std) of different methods on ORL dataset with a different percent of labeled data.

*ξ*	10%			20%			30%			40%		
	ACC	NMI	Purity	ACC	NMI	Purity	ACC	NMI	Purity	ACC	NMI	Purity
SC (1)	16.01 ± 0.55	37.19 ± 0.81	17.00 ± 0.67	16.00 ± 0.79	37.40 ± 0.74	17.06 ± 0.85	16.00 ± 0.61	37.51 ± 0.82	17.03 ± 0.79	16.00 ± 0.73	37.74 ± 0.58	16.97 ± 0.79
SC (2)	15.94 ± 0.51	37.64 ± 0.83	16.84 ± 0.61	16.24 ± 0.64	37.73 ± 0.72	17.07 ± 0.73	16.35 ± 0.57	37.86 ± 0.73	17.39 ± 0.74	16.32 ± 0.57	37.73 ± 0.93	17.19 ± 0.65
SC (3)	16.51 ± 0.55	39.28 ± 0.66	17.22 ± 0.66	16.24 ± 0.70	39.07 ± 0.67	17.00 ± 0.81	16.73 ± 0.72	39.66 ± 0.89	17.32 ± 0.83	16.45 ± 0.74	39.37 ± 0.83	17.30 ± 0.93
SC (concat)	14.92 ± 2.93	34.22 ± 5.96	16.35 ± 2.53	15.05 ± 2.27	34.99 ± 4.38	16.22 ± 2.00	14.43 ± 2.98	33.09 ± 6.10	15.65 ± 2.27	14.60 ± 3.07	33.34 ± 6.26	15.90 ± 2.44
MVSC	28.27 ± 1.89	48.13 ± 1.71	29.82 ± 1.87	36.54 ± 2.26	54.06 ± 1.42	37.48 ± 2.04	42.01 ± 2.30	57.98 ± 1.50	42.94 ± 1.99	47.76 ± 2.17	60.50 ± 1.23	48.11 ± 1.96
AMGL	79.85 ± 1.27	89.72 ± 0.74	81.15 ± 1.24	83.11 ± 1.92	91.17 ± 0.86	84.39 ± 1.55	85.35 ± 1.84	92.10 ± 0.80	86.10 ± 1.30	83.81 ± 2.36	91.52 ± 1.12	85.03 ± 2.00
MLAN	67.19 ± 1.55	82.06 ± 0.92	71.84 ± 1.41	69.17 ± 1.04	82.78 ± 0.55	73.11 ± 0.66	70.47 ± 1.23	83.08 ± 0.54	73.84 ± 0.86	70.67 ± 0.89	83.16 ± 0.52	73.91 ± 0.59
SMVC_WAGE	**84.97** ± **2.25**	**89.73** ± **1.51**	**85.00** ± **2.26**	**94.44** ± **1.14**	**95.94** ± **0.85**	**94.44** ± **1.14**	**97.45** ± **0.89**	**98.00** ± **0.62**	**97.45** ± **0.89**	**98.69** ± **0.76**	**98.97** ± **0.55**	**98.69** ± **0.76**

Bold numbers denote the best results.

**Table 5:** Aggregated ACC (%), NMI (%), and Purity (%) comparison (mean ± std) of different methods on NUS-WIDE-OBJECT dataset with a different percent of labeled data.

*ξ*	10%			20%			30%			40%		
	ACC	NMI	Purity	ACC	NMI	Purity	ACC	NMI	Purity	ACC	NMI	Purity
SC (1)	18.84 ± 1.02	0.52 ± 0.10	27.12 ± 0.29	18.93 ± 1.27	0.57 ± 0.11	27.25 ± 0.29	18.49 ± 0.92	0.52 ± 0.11	27.06 ± 0.23	18.47 ± 1.01	0.53 ± 0.10	27.15 ± 0.26
SC (2)	18.58 ± 0.68	0.71 ± 0.18	27.20 ± 0.28	18.64 ± 0.77	0.68 ± 0.18	27.21 ± 0.26	18.58 ± 0.77	0.76 ± 0.19	27.20 ± 0.34	18.39 ± 0.63	0.70 ± 0.20	27.20 ± 0.33
SC (3)	20.65 ± 0.06	2.27 ± 0.10	28.09 ± 0.14	20.67 ± 0.12	2.22 ± 0.08	28.11 ± 0.24	20.65 ± 0.09	2.21 ± 0.12	28.16 ± 0.25	20.61 ± 0.11	2.20 ± 0.13	28.13 ± 0.22
SC (4)	17.70 ± 0.31	0.78 ± 0.08	27.46 ± 0.24	17.78 ± 0.27	0.79 ± 0.08	27.34 ± 0.28	17.83 ± 0.30	0.77 ± 0.06	27.29 ± 0.26	17.77 ± 0.33	0.75 ± 0.07	27.32 ± 0.26
SC (5)	19.50 ± 1.07	1.22 ± 0.47	27.23 ± 0.38	19.79 ± 1.07	1.27 ± 0.36	27.08 ± 0.22	19.50 ± 0.99	1.26 ± 0.37	27.17 ± 0.29	19.44 ± 0.93	1.19 ± 0.37	27.10 ± 0.17
SC (concat)	18.17 ± 0.55	0.91 ± 0.33	27.30 ± 0.42	18.29 ± 0.72	0.93 ± 0.26	27.17 ± 0.36	18.31 ± 0.89	0.95 ± 0.29	27.15 ± 0.48	18.60 ± 0.74	0.95 ± 0.29	27.17 ± 0.32
MVSC	17.36 ± 0.24	0.38 ± 0.05	26.94 ± 0.02	16.87 ± 0.12	0.34 ± 0.03	26.93 ± 0.00	16.63 ± 0.28	0.25 ± 0.03	26.93 ± 0.00	17.06 ± 0.25	0.26 ± 0.04	26.93 ± 0.00
AMGL	27.03 ± 0.46	6.79 ± 0.15	29.79 ± 0.43	27.17 ± 0.52	6.79 ± 0.11	30.09 ± 0.70	26.89 ± 0.50	6.74 ± 0.11	29.71 ± 0.41	27.07 ± 0.55	6.77 ± 0.12	29.82 ± 0.41
MLAN	26.85 ± 0.03	6.17 ± 0.15	27.43 ± 0.00	26.88 ± 0.08	6.15 ± 0.16	27.41 ± 0.06	26.90 ± 0.00	6.42 ± 0.00	27.57 ± 0.00	26.90 ± 0.00	6.40 ± 0.03	27.57 ± 0.00
SMVC_WAGE	**38.05** ± **1.43**	**13.30** ± **0.92**	**40.44** ± **1.00**	**40.13** ± **1.33**	**14.29** ± **0.71**	**41.19** ± **0.89**	**40.37** ± **1.64**	**14.49** ± **0.78**	**41.63** ± **0.94**	**40.74** ± **1.09**	**14.59** ± **0.59**	**41.67** ± **0.60**

Bold numbers denote the best results.

**Table 6:** Aggregated ACC (%), NMI (%), and Purity (%) comparison (mean ± std) of different methods on MSRC-v1 dataset with a different percent of labeled data.

*ξ*	10%			20%			30%			40%		
	ACC	NMI	Purity	ACC	NMI	Purity	ACC	NMI	Purity	ACC	NMI	Purity
SC (1)	27.00 ± 2.54	11.11 ± 2.45	28.17 ± 2.35	27.62 ± 1.83	10.89 ± 2.44	28.52 ± 1.76	27.45 ± 2.19	11.29 ± 2.17	28.57 ± 2.37	26.76 ± 1.77	10.94 ± 2.40	27.88 ± 2.13
SC (2)	74.74 ± 1.57	59.47 ± 2.18	74.74 ± 1.57	75.88 ± 1.30	60.74 ± 1.50	75.88 ± 1.30	76.10 ± 1.28	60.80 ± 1.59	76.10 ± 1.28	76.10 ± 1.35	60.82 ± 1.75	76.10 ± 1.35
SC (3)	80.57 ± 2.74	69.41 ± 2.02	80.76 ± 2.05	81.19 ± 2.75	70.33 ± 1.93	81.38 ± 2.00	81.95 ± 1.23	70.58 ± 1.97	81.95 ± 1.23	82.31 ± 1.00	71.09 ± 1.61	82.31 ± 1.00
SC (4)	32.19 ± 3.59	17.23 ± 3.31	33.67 ± 3.38	31.69 ± 2.93	18.50 ± 2.93	33.93 ± 3.05	30.45 ± 2.52	16.54 ± 3.15	32.12 ± 2.64	32.43 ± 2.80	16.74 ± 2.66	33.74 ± 2.78
SC (5)	62.74 ± 2.70	48.63 ± 1.72	64.10 ± 1.97	64.36 ± 1.27	49.71 ± 1.47	65.26 ± 1.23	64.55 ± 1.12	49.86 ± 1.46	65.45 ± 0.98	64.86 ± 0.81	50.19 ± 1.16	65.74 ± 0.75
SC (concat)	78.71 ± 2.29	69.88 ± 2.53	78.86 ± 2.01	79.57 ± 1.68	70.79 ± 2.17	79.71 ± 1.39	79.81 ± 1.44	70.82 ± 2.29	79.81 ± 1.44	80.29 ± 1.42	71.68 ± 1.96	80.29 ± 1.42
MVSC	46.86 ± 3.52	32.69 ± 2.73	48.38 ± 3.35	46.98 ± 1.62	31.39 ± 1.36	48.07 ± 1.83	47.64 ± 2.93	32.38 ± 2.18	50.33 ± 2.92	44.48 ± 0.92	27.35 ± 0.97	47.05 ± 1.39
AMGL	86.00 ± 2.55	**77.89** ± **2.07**	86.00 ± 2.55	85.74 ± 2.26	77.35 ± 2.06	85.74 ± 2.26	86.76 ± 2.34	78.41 ± 2.21	86.76 ± 2.34	87.12 ± 2.28	78.87 ± 2.20	87.12 ± 2.28
MLAN	68.10 ± 0.00	66.24 ± 0.00	73.33 ± 0.00	68.36 ± 1.17	66.14 ± 0.44	73.33 ± 0.00	68.10 ± 0.00	66.24 ± 0.00	73.33 ± 0.00	68.10 ± 0.00	66.24 ± 0.00	73.33 ± 0.00
SMVC_WAGE	**87.40** ± **3.16**	77.29 ± 3.70	**87.40** ± **3.16**	**91.17** ± **1.87**	**82.73** ± **3.19**	**91.17** ± **1.87**	**92.57** ± **1.38**	**85.11** ± **2.59**	**92.57** ± **1.38**	**93.36** ± **1.39**	**86.69** ± **2.44**	**93.36** ± **1.39**

Bold numbers denote the best results.

**Table 7:** Aggregated ACC (%), NMI (%), and Purity (%) comparison (mean ± std) of different methods on 3Sources dataset with a different percent of labeled data.

*ξ*	10%			20%			30%			40%		
	ACC	NMI	Purity	ACC	NMI	Purity	ACC	NMI	Purity	ACC	NMI	Purity
SC (1)	27.76 ± 2.18	5.83 ± 1.72	30.24 ± 1.84	26.61 ± 2.11	5.58 ± 1.58	29.36 ± 1.69	27.34 ± 1.95	5.44 ± 1.78	29.41 ± 2.08	27.78 ± 2.40	6.38 ± 1.66	30.78 ± 1.97
SC (2)	24.18 ± 1.25	3.65 ± 0.82	27.38 ± 1.38	24.82 ± 1.79	4.04 ± 0.77	27.69 ± 1.21	24.77 ± 1.77	3.82 ± 1.43	28.06 ± 1.77	24.96 ± 1.39	3.90 ± 0.90	27.82 ± 1.17
SC (3)	27.96 ± 2.11	5.22 ± 1.15	30.84 ± 1.62	27.69 ± 2.61	4.99 ± 1.31	30.78 ± 2.09	27.30 ± 2.47	5.01 ± 0.98	30.65 ± 1.50	27.84 ± 2.70	5.19 ± 1.13	31.14 ± 1.97
SC (concat)	22.90 ± 0.76	2.38 ± 0.47	26.48 ± 0.83	23.28 ± 1.51	2.56 ± 0.82	27.16 ± 0.98	23.02 ± 1.33	2.39 ± 0.80	26.86 ± 1.11	22.96 ± 1.28	2.20 ± 0.64	26.41 ± 0.80
PVC (V1–V3)	26.04 ± 0.00	5.63 ± 0.00	26.54 ± 0.00	26.04 ± 0.00	5.63 ± 0.00	26.54 ± 0.00	26.04 ± 0.00	5.63 ± 0.00	26.54 ± 0.00	26.04 ± 0.00	5.63 ± 0.00	26.54 ± 0.00
IMG (V1–V3)	68.12 ± 1.91	57.60 ± 0.53	68.27 ± 1.67	66.88 ± 0.88	57.45 ± 0.24	67.08 ± 0.54	69.00 ± 1.33	58.00 ± 0.48	69.10 ± 1.14	68.87 ± 1.43	57.96 ± 0.59	68.92 ± 1.29
DAIMC	66.90 ± 0.36	54.28 ± 0.35	73.15 ± 0.36	62.68 ± 1.40	46.82 ± 0.45	63.15 ± 0.70	79.74 ± 0.37	60.05 ± 0.46	79.74 ± 0.37	71.83 ± 0.35	57.55 ± 0.37	71.83 ± 0.35
IMSC_AGL	81.59 ± 0.65	69.47 ± 0.73	81.59 ± 0.65	81.73 ± 0.00	69.63 ± 0.00	81.73 ± 0.00	81.59 ± 0.65	69.47 ± 0.73	81.59 ± 0.65	81.73 ± 0.00	69.63 ± 0.00	81.73 ± 0.00
APMC	85.34 ± 0.00	71.18 ± 0.18	85.34 ± 0.00	85.34 ± 0.00	71.13 ± 0.17	85.34 ± 0.00	85.34 ± 0.00	71.14 ± 0.17	85.34 ± 0.00	85.34 ± 0.00	71.10 ± 0.06	85.34 ± 0.00
SMVC_WAGE	**88.94** ± **1.71**	**75.87** ± **2.71**	**88.94** ± **1.71**	**92.14** ± **1.11**	**81.90** ± **2.31**	**92.14** ± **1.11**	**93.16** ± **0.70**	**83.98** ± **1.67**	**93.16** ± **0.70**	**93.68** ± **0.46**	**85.05** ± **1.05**	**93.68** ± **0.46**

Bold numbers denote the best results.

**Table 8:** Aggregated comparison (mean ± std) of the average running time with a different percent of labeled data in different methods on six real-world datasets (in seconds).

Complete data clustering								

Datasets	SC (best)	SC (concat)	MVSC	AMGL	MLAN	SMVC_WAGE	—	—
Cornell	0.32 ± 0.01	0.47 ± 0.01	0.44 ± 0.03	0.37 ± 0.01	0.24 ± 0.03	**0.23** ± **0.02**	—	—
Digit	1.45 ± 0.02	9.72 ± 0.13	14.57 ± 0.16	62.73 ± 1.55	28.56 ± 2.40	**0.36** ± **0.03**	—	—
ORL	5.56 ± 0.11	22.31 ± 0.31	3.96 ± 0.23	0.64 ± 0.01	1.15 ± 0.11	**0.40** ± **0.03**	—	—
NUS	6.88 ± 0.09	23.10 ± 0.10	29.96 ± 0.64	180.78 ± 1.02	71.67 ± 8.00	**0.41** ± **0.04**	—	—
MSRC-v1	**0.10** ± **0.00**	0.35 ± 0.09	0.42 ± 0.02	0.26 ± 0.01	0.32 ± 0.04	0.28 ± 0.03	—	—

Incomplete data clustering								

Datasets	SC (best)	SC (concat)	PVC (V1–V3)	IMG (V1–V3)	DAIMC	IMSC_AGL	APMC	SMVC_WAGE
3Sources	3.16 ± 0.09	16.85 ± 0.41	1.25 ± 0.10	18.74 ± 0.32	262.61 ± 2.32	52.56 ± 1.89	0.63 ± 0.19	**0.37** ± **0.01**

All experiments are conducted on a PC machine with an Intel(R) Core(TM) i7-5557U CPU @ 3.10 GHz and 16 G RAM in the MATLAB environment. Bold numbers denote the best results.

## Data Availability

Six publicly available benchmark multi-view datasets are utilized: the Cornell dataset, 3Sources dataset, UCI Handwritten Digit dataset, ORL dataset, NUS-WIDE-OBJECT dataset, and MSRC-v1 dataset. All the multi-view datasets' homepages are listed in this paper.
